The article "Medication Regularity of Traditional Chinese Medicine in the Treatment of Aplastic Anemia Based on Data Mining" was published in 2022. Journal: Evid Based Complement Alternat Med.

# Medication Regularity of Traditional Chinese Medicine in the Treatment of Aplastic Anemia Based on Data Mining

**DOI:** 10.1155/2022/1605359

**Published:** 2022-08-25

**Authors:** Nanxi Dong, Xujie Zhang, Dijiong Wu, Zhiping Hu, Wenbin Liu, Shu Deng, Baodong Ye

**Affiliations:** ^1^The First School of Clinical Medicine, Zhejiang Chinese Medical University, Hangzhou, China; ^2^The College of Control Science and Engineering, Zhejiang University, Hangzhou, China

## Abstract

**Objective:**

Aplastic anemia (AA) is an uncommon disease, characterized by pancytopenia and hypocellular bone marrow, but it is common in the blood system. The medication rules of traditional Chinese medicine (TCM) in the treatment of AA are not clear, for which it is worth exploring the medication rules by data mining methods.

**Methods:**

This study used SPSS Modeler 18.0 and SPSS statistics to analyze the cases of AA from Zhejiang Provincial Hospital of Chinese Medicine (ZJHCM) from March 1, 2019, to March 1, 2022. Data mining methods, including frequency analysis, cluster analysis, and association rule learning, were performed in order to explore the medication rules for AA.

**Results:**

(1) A total of 859 prescriptions, which met the inclusion criteria, consisted of 255 herbs. In descending order of the frequency of herbal medicine, we have Danggui, Huangqi, Shudihuang, Fuling, Gancao, Shanyao, Shanzhuyu, Baizhu, Dangshen, and Xianhecao. (2) Frequency analysis of herb properties: the Four Qi of 255 kinds of TCMs are mainly warm and neutral medicines. The Five Flavors are mainly sweet medicines, followed by bitter medicines. The main meridians are the liver, spleen, and kidney. (3) Clustering of medications: TCMs with the top 20 frequencies are classified into 9 groups by cluster analysis. (4) Association rule analysis of high-frequency herbs: using the Apriori algorithm, the results showed that there were 3 herb pairs with support of over 0.3 and 12 herb pairs with confidence above 0.85.

**Conclusion:**

The basic pathogenesis of AA (Sui Lao) is spleen and kidney essence deficiency, Qi deficiency, and blood stasis. The main herbs have warm and neutral properties, sweet tastes, and liver, spleen, and kidney meridian tropisms, whose purpose is to tonify the kidney and invigorate the spleen, tonify Qi, and promote blood circulation.

## 1. Introduction

Aplastic anemia (AA) is a disease associated with bone marrow failure, which is mainly characterized by pancytopenia and infection due to decreased hematopoiesis in bone marrow [1, 2]. Patients with AA usually have a poor quality of life and high economic pressure. The treatment methods for AA include immunosuppressive therapy (IST), allogeneic hematopoietic stem cell transplantation (allo-HSCT), and supportive care [3]. Among patients who received first-line IST, 10-year overall survival (OS) and failure-free survival (FFS) rates were 55% and 40%, respectively [4]. In the National Institutes of Health (NIH) clinical trial of treating with IST, approximately one-third of responding patients, either relapsed or required sustained cyclosporine administration to maintain their blood counts [5]. 30%–40% of patients showed no response to treatment with antithymocyte globulin (ATG), which will also consume platelets. Allo-HSCT is considered as the first-line treatment for young and adult patients who may have an HLA-matched sibling donor (MSD) [6–8]. A study conducted by the Severe Aplastic Anemia Working Party of the European Society for Blood and Marrow Transplantation (SAAWP-EBMT) showed that graft-versus-host disease-free, relapse-free survival (GRFS) of allo-HSCT for AA was only 69% over 5 years [9]. However, the remaining patients still have complications, such as graft-versus-host disease (GVHD) [10], virus infection [11], poor graft function [12], and so on. Although the treatment of AA in Western medicine is developing rapidly, there are still many nonnegligible clinical symptoms. With these treatments in patients with AA, the 5-year survival rate approaches 60–80% [13, 14]. A switch to a second-line regimen is recommended when there is treatment failure with first-line treatments. However, patients may face not only higher medical expenditure but also higher medical risk. In addition, the transfusion support will lead to a risk of iron overload [15–17]. Therefore, according to the different treatment stages of patients, the combination therapy of TCM is a common trend. The treatment strategies by integrative medicine could reduce the side effects and complications. It is noted that traditional Chinese medicine (TCM) treatment of AA medication rules is not clear, so it is necessary to carry out data mining on TCM treatment of AA.

The article "Medication Regularity of Traditional Chinese Medicine in the Treatment of Aplastic Anemia Based on Data Mining" was published in 2022. Journal: Evid Based Complement Alternat Med.

The name “aplastic anemia” does not appear in the ancient Chinese classics, whose clinical manifestations tend to be “consumptive disease” or “hemorrhagic syndrome” in traditional Chinese concepts [18]. In the 1950s, AA was thought to be a deficiency of Qi and blood according to the clinical manifestations of the patients [19]. In the 1960s, on the basis of the syndrome differentiation of Qi and blood, the effects of Guipi Decoction and Bazhen Decoction were poor [20]. In the 1970s, according to the syndrome differentiation of yin and yang of viscera, the focus was shifted from the heart and spleen to the liver and kidney, and the efficacy of Zuoguiyin and Youguiyin in the treatment of AA was improved [21, 22]. In 1989, the Dalian National Symposium on Hematology of Integrated Traditional Chinese and Western Medicine associated the classification of AA with the kidney, which was analyzed by syndrome differentiation methods of zang-fu viscera and eight principles. Chronic aplastic anemia belongs to consumptive disease and blood insufficiency, which can be divided into kidney yin deficiency, kidney yang deficiency, and deficiency of both kidney yin and yang [21, 23]. In 2008, the China Association of Chinese Medicine issued guidelines for the diagnosis and treatment of common diseases in Chinese medicine, where the syndromes of spleen-kidney yang deficiency, liver-kidney yin deficiency, heat-toxin congestion, and blood heat syndrome were added [24]. In recent years, TCM has gained increasing attention in AA therapy. A previous study has shown that the hemocyte profile in the Shenlu granule combined treatment group was superior to the therapeutic effect in the western medicine alone group based on kidney reinforcing syndrome [25]. Another study suggested that potential mechanisms of Siwu Paste are to improve hematopoietic microenvironment and promote bone marrow hematopoiesis therapies [26]. However, these treatments are still limited in clinical application.

With the popularity of medical informatization, a large amount of medical data can be collected, stored, and analyzed, which also promotes the development of data mining in the medical field. Data mining technology [27] is a decision support process that can analyze data automatically, inductive reasoning, and mine potential patterns. The computer-based data mining technology employs algorithms to extract latent information embedded in a large amount of medical data and provides valuable guidance for the treatment of diseases. At present, data mining can complete many tasks, mainly including association analysis, cluster analysis, classification, prediction, and so on [28], which makes it applicable to scenarios such as symptom and sign analysis [29], syndrome differentiation [30], and medication rule analysis [31]. To explore the medication rules for AA and provide integrated TCM-based treating suggestions, 859 prescriptions were adopted to obtain the medication rules from high-frequency Chinese medicine, Four Qi and Five Flavors of TCM, and their meridian tropism.

The treatment of AA in ZJHCM is characterized by integrated TCM and Western medicine. We also paid attention to adjusting zang-fu viscera, especially in kidney and spleen, and Qi, blood, and water. It is reported by ZJHCM that compared with treated with IST alone, standard IST for severe aplastic anemia (SAA) could improve hematologic responses, bone marrow hyperplasia, and clinical symptoms. [32]. It is also reported that treatment with the TCM may reduce the rate of graft failure and treatment-related mortality and improve the rate of (overall survival) OS in SAA patients with allo-HSCT [18]. Besides, a study revealed the TCM of Bushen Jianpi Quyu Formula in AA could alleviate myelosuppression by inhibiting the expression of the PI3K/AKT/NF-*κ*B signaling pathway [33]. It is a strong benefit for patients in various ways by TCM. However, research about current treatment patterns of AA in China reported that among the 352 enrolled patients, 43 patients (12.6% of all) received TCM, and only 3 of them used TCM as the main treatment regimen for AA [34]. Therefore, we analyzed the characteristics of TCM treatment of AA in ZJHCM by data mining.

The article "Medication Regularity of Traditional Chinese Medicine in the Treatment of Aplastic Anemia Based on Data Mining" was published in 2022. Journal: Evid Based Complement Alternat Med.

## 2. Materials and Methods

Data mining can be composed of three main stages: first, data cleaning is performed on the collected data, which could remove noisy data so that the model can obtain more representative conclusions; next, the processed high-quality dataset could be used to construct a model, which extracts the relationship between the data; and finally, visualization technology can intuitively display the potential information extracted by the model, which is helpful for decision-makers to summarize and analyze.

### 2.1. Data Source and Processing

This study adopted a total of 1263 cases of AA from ZJHCM from March 1, 2019 to March 1, 2022. Including criteria are as follows: (1) compliance with diagnostic criteria for AA, (2) a complete TCM treatment prescription with at least one revisit. Excluding criteria are as follows: (1) patients with severe liver and kidney dysfunction, (2) TCM for external use, (3) prescriptions with more than 10 visits for the same patient, and (4) patients after HSCT and IST treatment. The screening process results in 859 prescriptions being collected. The herb names were standardized, where Shenghuangqi and Zhihuangqi were unified as Huangqi, as well as Shenggancao and Zhigancao were unified as Gancao, and the information of properties, tastes, and meridian tropisms was complemented according to Chinese pharmacopoeia [35].

Some of the collected prescriptions are shown in Table 1, which need to be processed by *Python* to make them conform to the input form of SPSS. Then the prescriptions for a single visit were integrated, which obtained 859 prescriptions, involving 255 kinds of TCMs (Table 2). Finally, an all-zero matrix is created with the column name of the herb name, and its sparse matrix form (Table 3) is obtained by *Python* according to the integrated prescription (Table 2).

The article "Medication Regularity of Traditional Chinese Medicine in the Treatment of Aplastic Anemia Based on Data Mining" was published in 2022. Journal: Evid Based Complement Alternat Med.

### 2.2. Frequency Analysis

Frequency analysis is a typical analytical method of descriptive statistics, which can be utilized to describe the statistical values of variables. Frequency analysis for TCMs has been widely used to extract prescription rules and to provide the basis for clinical forecasting and decision-making. It is beneficial to better understand the nature of diseases and the typical methods of prevention or treatment. To analyze the characteristics of AA and to explore the preference of its herbal treatment, frequency analysis was applied to study the frequency of occurrence, properties, tastes, and meridian tropisms of all TCM involved. All frequency analyses were performed in Microsoft Excel 2016. The frequency of herbal medicine is calculated as follows:

(1) $$\begin{array}{c} \text{frequency}\left(a\right)=\left(\frac{a}{b}\right)\times 100\%, \end{array}$$

where *a* means the usage times of a particular herbal medicine and *b* denotes the total number of prescriptions.

### 2.3. Cluster Analysis

As an important part of unsupervised learning, cluster analysis can automatically classify a variety of objects, such as herbs, with the same nature from the data itself when the category of objects is unknown. In the field of research on medication rules, cluster analysis can classify various medicinal materials into regular groups, so as to reveal the potential combination rules of prescriptions. In order to discover and summarize reasonable herbal combinations for the treatment of AA, cluster analysis of the top 40 herbs was carried out by utilizing IBM SPSS Statistics. The hierarchical cluster method based on Pearson correlation coefficient was chosen as the data mining method to obtain cluster results with the calculated values standardized by Z scores for comparison [30]. Finally, the clustering results are displayed in the form of a dendrogram.

The calculation scheme of the hierarchical cluster method based on the Pearson correlation coefficient is offered as follows:

1. Set each sample as one class and calculate the Pearson distance between each two classes
2. Find the nearest two classes between each class and merge them into one class to reduce the total number of classes
3. Recalculate the similarity between the newly generated class and each old class
4. Repeat steps 2 and 3 until all sampling points are divided into 9 categories

The Pearson correlation coefficient is used to calculate the relationship between two variables *X* and *Y* as follows:

(2) $$\begin{array}{c} \rho_{X,\;Y}=\frac{\sum_{i=1}^{n}x_{i}y_{i}-\left(\sum_{i=1}^{n}x_{i}\right)\times \left(\sum_{i=1}^{n}y_{i}\right)/n}{\sqrt{\left.\left(\sum_{i=1}^{n}x_{i}^{2}\right)-{\left(\sum_{i=1}^{n}x_{i}\right)}^{2}/n\right)\times \left.\left(\sum_{i=1}^{n}y_{i}^{2}\right)-{\left(\sum_{i=1}^{n}y_{i}\right)}^{2}/n\right)}}, \end{array}$$

where *X*=(*x*_1_, *x*_2_,  *x*_3_ …,  *x*_*n*_) and *Y*=(*y*_1_, *y*_2_,  *y*_3_ …,  *y*_*n*_). The correlation coefficient ranges from [−1,1], where the value 1 represents a perfect correlation, value 0 means no correlation, and value −1 represents negative correlation.

The article "Medication Regularity of Traditional Chinese Medicine in the Treatment of Aplastic Anemia Based on Data Mining" was published in 2022. Journal: Evid Based Complement Alternat Med.

### 2.4. Association Rule Analysis

Association rule analysis is an unsupervised learning method, which reveals the internal structure of a dataset. It was first proposed to discover the relationship between different commodities in supermarket sales data to make better sales plans. In the study of medication rules, association rule analysis can also be used to explore the co-occurrence rules between herbs. To explore combinatorial rules for the treatment of AA, an SPSS modeler was adopted to perform association rule learning for all herbs in this study. The Apriori algorithm is chosen to obtain candidate item sets [36], where support and confidence are used to select important rules. The Apriori algorithm is chosen to obtain candidate item sets [37], where support and confidence are used to select important rules. Support refers to the probability that an itemset appears in all item sets. A high support value means that this association rule is very significant. Confidence is the ratio of the frequency that the antecedent and consequent items cooccur to the frequency that the antecedent item occurs individually, indicating the accuracy of the rule [38]. The support and confidence of rule is expressed as follows:

(3) $$\begin{array}{c} \mathrm{support}\left(x⟶y\right)=\mathrm{support}\;\left(X\cup^{\;}\;Y\right)=\frac{\text{count }\left(X\cup^{\;}Y\right)}{\text{count}\left(D\right)},\\ \text{confidence }\left(X\cup^{\;}\;Y\right)=\frac{\text{support }\left(X\;\cup^{\;}\;Y\right)}{\text{support }\left(X\right)},\\ \text{lift }\left(X⟶Y\right)=\;\frac{\text{confidence}\left(X\;⟶\;Y\right)}{\text{support}\left(Y\right)}. \end{array}$$

X and Y are examples of associations represented by association rules. For example, *X*=herb 1 and *Y*=*herb* 1, and *X*∩^ ^ *Y*=herb 1 are the set of all items in D. If the percentage of *X* ∪^ ^ *Y* in the dataset D is a%, then the support of the association rule *X*⟶*Y* is a%. In fact, the support is a probability value. The lift is the ratio of the probability of item Y appearing in the presence of X to the frequency of Y. Support and confidence are often used to eliminate meaningless combinations, and lift could show the validity of the rules.

The article "Medication Regularity of Traditional Chinese Medicine in the Treatment of Aplastic Anemia Based on Data Mining" was published in 2022. Journal: Evid Based Complement Alternat Med.

To extract more representative rules, the minimum threshold of support was set to 0.20 and the minimum value of confidence was set to 0.8. Besides, the maximum number of antecedent items was set to 2.

## 3. Results

### 3.1. Frequency Analysis

#### 3.1.1. Medication Frequency

After data collection and processing, the frequency of herbal medicine use (Figure 1) was calculated, involving a total of 255 herbs in 859 prescriptions. In this study, herbal medicines were ranked from high to low according to the usage frequency, and the cumulative total frequency of herb use was 16129. As shown in Figure 1, the top 10 most commonly used herbs were: Danggui (602 times, 70.08%), Huangqi (599 times,69.73%), Shudihuang (539 times, 62.75%), Fuling (493 times, 57.39%), Gancao (469 times, 54.60%), Shanyao (437 times, 50,87%), Shanzhuyu (421 times, 49.01%), Baizhu (413 times, 48.08%), Dangshen (365 times, 42.49%), and Xianhecao (358 times, 41.68%). Most of them belong to tonics, and others have the effect of promoting blood circulation and eliminating dampness.

#### 3.1.2. Properties, Tastes, and Meridian Tropisms of Herbs

The medicinal properties of TCM are divided into Yin and Yang. The “Four Qi” of TCM are as follows: cold, hot, warm, and cool. Besides, herbs with moderate effects are mild. Five flavors of TCM refer to the taste of herbs, including sour, bitter, sweet, pungent, and salty, which are commonly known as the most basic tastes. In addition, they are weak, astringent, etc. In order to correspond to the theory of the five elements in imperial China, astringency was attached to the sour and weakness attached to the sweet, with which all of them could be called Five Flavors. A medicine meridian denotes the site of drug action. Medicine meridian matches the effect of herbs with the theory of viscera and meridians to illustrate the selectivity of drug action to a certain site of the body.

It can be shown in g (c) that the herb's meridian tropisms are ranked as liver, spleen, kidney, lung, heart, stomach, gallbladder, large intestine, bladder, small intestine, pericardium, and triple energizer in descending order based on the frequency. The frequency of herb's meridian tropisms above 15% are liver, spleen, and kidney.

Figure 2(a) and 2(b) describe the distribution of herbs' Four Qi and Five Flavors. In descending order of frequency, the Four Qi of the herb are arranged as: warm, mild, cold, cool, and hot. The occurrence of warm herbs was 6950 times, and its frequency was up to 43.83%, which was much higher than other medicinal properties. The frequencies of the Five Flavors are ranked as sweet, bitter, pungent, sour, astringent, weak, and salty from high to low, where sweet medicines accounted for 42.05% of the total.

The article "Medication Regularity of Traditional Chinese Medicine in the Treatment of Aplastic Anemia Based on Data Mining" was published in 2022. Journal: Evid Based Complement Alternat Med.

### 3.2. Cluster Analysis

The cluster analysis results of high-frequency herbs were obtained by SPSS statistics:

1. Most herbs of Group 1 can be used to invigorate the kidney, cool the blood, and stop bleeding, except Maiya
2. In Group 2, Baishao and Chuanxiong belong to Chinese traditional Siwu decoction, and it was described by the ancients that the effect of Danshen is equivalent to that of Siwu Decoction
3. Herbs of Group 3 have the effect of improving indigestion
4. Herbs of Group 4 can invigorate spleen to nourish original Qi
5. The goal of Group 5 is to tonify Qi and consolidate superficies
6. Group 9 is contributing to nourishing kidney essence

The first six categories are meaningful in clinical prescription, and the results are shown in Figure 3.

### 3.3. Association Rule Analysis

The results of association rule analysis can mine the combination of potential core herbs from commonly used prescriptions. The results showed that there were three herb combinations with support over of 30% (“Danggui-Jixueteng,” “Danggui-Yinyanghuo,” and “Huangqi-Fangfeng”), whose objective is mainly to nourish blood, activate blood, and tonify the kidneys and Qi (Table 4). From the constructed network diagram (Figure 4), it can be seen that Danggui, Huangqi, and Fuling are the core herbs for treating AA, which is consistent with the conclusion of frequency analysis.

## 4. Conclusion

AA is a bone marrow hematopoietic dysfunction disease called “Suilao” or “Consumptive disease” in TCM. The main clinical symptoms of AA are hypodynamia, hemorrhage, and infection. In our center, we treated AA by integrating traditional Chinese medicine and western medicine, to reduce the clinical symptoms of patients, improve their quality of life, and alleviate their economic burden.

Based on data mining, we studied the regularity of TCM for the treatment of AA in our center. The top three herbs are Danggui (602 times, 70.08%), Huangqi (599 times, 69.73%), and Shudihuang (539 times, 62.75%). In terms of TCM, Danggui can replenish blood and activate blood. Besides, Danggui has an immunomodulatory effect [39]. Huangqi can nourish Qi and promote water metabolism. In clinical practice, Huangqi could enhance the nonspecific immune function of organisms, regulate humoral immunity, and normalize cellular immunity [40]. Shudihuang has the effect of invigorating the kidneys. A study indicates that there is an influence of the “bone marrow system” by the “kidney marrow” in TCM [41]. According to the results, Fuling, Gancao, Shanyao, Shanzhuyu, Baizhu, Dangshen, and Xianhecao follow. It revealed that the basic principle of treatment in AA was to strengthen the liver and kidney, as well as nourish Qi and blood. Moreover, herbs that promote water metabolism are often added to prescriptions, eliminating dampness and promoting hematopoiesis.

The article "Medication Regularity of Traditional Chinese Medicine in the Treatment of Aplastic Anemia Based on Data Mining" was published in 2022. Journal: Evid Based Complement Alternat Med.

Ancient medical books called “Jingyue Quanshu” indicated that the therapy of TCM for patients with blood deficiency and stasis is enriching blood and promoting blood circulation, which is the origin of the method of Bushen Huoxue. According to experience, the Chinese medical pathogenesis of AA is generated by “deficiency”. However, it is found that “stasis” should be added to the pathogenesis. In our previous study [42], we found that the treatment of patients with AA can improve the engraftment of hematopoietic stem cell transplantation by kidney-reinforcing, blood-activating, and stasis-removing. It has been reported that BUSHEN HUOXUE decoction could reduce the expression of IL-6 [18], which might affect the stability of the hematopoietic microenvironment in bone marrow [43]. In addition, about 61% of patients with AA were complicated by syndromes of “blood stasis” [19]. In this study, the “Danggui-Jixueteng” combo showed the highest statistical support in association rule analysis, which may indicate that dispelling blood stasis is as important as tonifying the kidneys in treating AA. Nonetheless, eliminating the dampness had possessed similar pharmacologic or pharmacodynamic action of removing blood stasis [44]. Fuling and Huangqi can eliminate the dampness, which appears in high-frequency drugs or association analysis pairs. Based on the prescription management platform of ZJHCM, using SPSS statistics and SPSS modeling, this study adopts a variety of data mining methods, such as cluster analysis and association rule analysis, to explore and analyze the medical record. This study has summarized the Chinese medication rules for treating AA, which can facilitate TCM diagnosis, treatment, and experimental research and would be helpful for AA patients. The results of the above data mining process show that the basic principle of AA's therapeutic methods is strengthening kidney and liver, nourishing spleen Qi, and supplemented by the treatments of activating blood, and eliminating dampness. The focus of treatment is to improve the bone marrow microenvironment by tonifying the kidneys and promoting blood circulation. By analyzing Four Qi and Five Flavors of the sample herbs, we found out that sweet and warm are the top 2 most frequent properties, which could nourish Qi. However, heat-clearing herbs are also used when necessary. We focus on nourishing the liver, spleen, and kidney. The combination of Chinese and Western medicine in the treatment of AA alleviates the pain of patients. The conditions of patients change constantly, and we are continuing to explore and study.

The article "Medication Regularity of Traditional Chinese Medicine in the Treatment of Aplastic Anemia Based on Data Mining" was published in 2022. Journal: Evid Based Complement Alternat Med.

## Figures and Tables

**Figure 1:** Frequency chart of Chinese herbs treating Aplastic anemia (top 10).

**Figure 2:** Four Qi, Five Flavors, and herb's Meridian Tropisms (a) Four Qi. (b) Five Flavors. (c) Meridian tropism of herbs. Four Qi, Five Flavors, and Meridian tropism of herbs were analyzed by a radar chart in Microsoft Excel.

**Figure 3:** Results of cluster analysis.

**Figure 4:** Network Diagram of core herbs.

**Table 1:** Part of case prescriptions.

Date	No. (patient)	Herb name	Date	No. (patient)	Herb name
20190301	0001	Shengdihuang	20190304	0004	Bajitian
20190301	0001	Niuxi	20190304	0004	Cebaiye
20190301	0001	Shihu	20190304	0004	Guya

	……			……	
20190302	0002	Dangshen	20190304	0005	Baishao
20190302	0002	Baizhu	20190304	0005	Buguzhi
20190302	0002	Gancao	20190304	0005	Honghua

	……			……	
20190302	0003	Guizhi	20190304	0006	Shengshaishen
20190302	0003	Fuling	20190304	0006	Fuling
20190302	0003	Zexie	20190304	0006	Ganjiang

	……			……	

**Table 2:** Integrated prescriptions.

No. (prescription)	Herb 1	Herb 2	Herb 3	Herb 4	Herb 5	Herb 6	…
1	Shengdihuang	Niuxi	Shihu	Fangfeng	Dangshen	Danshen	…
2	Dangshen	Baizhu	Gancao	Danggui	Chenpi	Shanyao	…
3	Guizhi	Fuling	Zexie	Danshen	Longgu	Muli	…
4	Bajitian	Cebaiye	Guya	Biejia	Houpo	Taizishen	…
5	Baishao	Buguzhi	Honghua	Dangshen	Jixueteng	Taizishen	…
6	Shengshaishen	Fuling	Ganjiang	Gancao	Heshouwu	Baishao	…
7	Dangshen	Danggui	Honghua	Danshen	Taoren	Shengdihuang	…
8	Dangshen	Baizhu	Shudihuang	Danggui	Chaihu	Shanyao	…
9	Baishao	Shudihuang	Heshouwu	Danggui	Shanzhuyu	-	…
			……				

**Table 3:** Sparse matrix form of prescriptions.

No. (prescription)	Danggui	Huangqi	Fuling	Gancao	Shanyao	…
1	1	1	1	1	0	…
2	1	0	1	1	1	…
3	0	0	1	1	0	…
4	0	1	1	0	0	…
5	1	1	0	1	0	…
6	0	0	1	1	0	…
7	0	0	0	1	1	…

**Table 4:** Association rules.

No.	Consequent	Antecedent	Support (%)	Confidence (%)	Lift
1	Danggui	Jixueteng	36.06	80.26	1.172
2	Danggui	Yinyanghuo	33.72	82.70	1.207
3	Huangqi	Fangfeng	32.79	83.99	1.23
4	Danggui	Jixueteng, Huangqi	28.00	80.00	1.168
5	Shudihuang	Xianhecao, Shanzhuyu	27.65	80.17	1.532
6	Danggui	Xianhecao, Shanzhuyu	27.65	80.59	1.177
7	Shanzhuyu	Xianhecao, Shudihuang	26.72	82.97	1.689
8	Danggui	Xianhecao, Shudihuang	26.72	84.72	1.199
9	Fuling	Dangshen, Baizhu	26.02	81.61	1.436
10	Shudihuang	Yinyanghuo, Shanzhuyu	25.90	80.63	1.532
11	Danggui	Yinyanghuo, Shanzhuyu	25.90	86.04	1.256
12	Shanzhuyu	Yinyanghuo, Shudihuang	24.39	85.65	1.195
13	Danggui	Yinyanghuo, Shudihuang	24.39	84.69	1.221
14	Danggui	Jixueteng, Shudihuang	24.04	83.01	1.216
15	Danggui	Buguzhi, Shanzhuyu	23.69	80.79	1.179
.	Danggui	Baishao, Gancao	22.99	80.71	1.178
17	Shudihuang	Heshouwu	22.87	90.82	1.577
18	Danggui	Heshouwu	22.87	83.67	1,222
19	Shudihuang	Jixueteng, Xianhecao	22.64	80.41	1.467
20	Danggui	Jixueteng, Xianhecao	22.64	87.11	1.272
